# Achievement of sustainable environment through effectiveness of social media in Z generation of China

**DOI:** 10.1371/journal.pone.0292403

**Published:** 2023-11-15

**Authors:** Bing Chen, Ghulam Rasool Madni

**Affiliations:** 1 School of Marxism, DongGuan University of Technology, Dongguan, 523000, Guangdong, China; 2 Department of Economics, Division of Management and Administrative Science, University of Education, Lahore, Pakistan; Southeast University, BANGLADESH

## Abstract

Social media is emerged as a powerful communication tool over the past ten years. The Z generation’s green buying habits and purchase intentions are being reshaped by social media, which is helping to advance the development of a sustainable environment. The consumption of non-organic products has raised carbon emissions, so changing consumption patterns and purchase intentions is necessary for a more sustainable future. Moreover, earlier literature has the absence of a comprehensive behavior change model that explains the mechanism through which social media influences sustainable behaviors This study explores that how social media affects patterns of consumption for Z generation of China while considering the role of environmental concerns, subjective norms, eco-branding and eco-labeling on the basis of theory of planned behavior. A questionnaire is used to get information from the 563 Z generation respondents of China. The data is analyzed using Smart-PLS and empirical outcomes show that social media has a statistically significant influence on shaping and affecting green consumption behavior of China’s Z generation because it has the potential to reach a vast audience and spread awareness about environmental issues, leading to increased intention towards a sustainable environment and reduction in carbon emissions. It also provides a platform for individuals to express their opinions and engage in discussions on environmental issues. These developments are promising for the future of environmental sustainability as they indicate a growing interest in preserving the planet among the Z generation of China. It can be recommended as a policy tool that government and other organizations should support the development of informative content on social media platforms, highlighting the importance of environmental sustainability and eco-friendly habits.

## 1. Introduction

The promotion of socio-economic models is an outcome of the urgent need to protect the environment due to limited natural resources. Now organizations are evolving into collaborative and open environments where new "distinctive" knowledge is developed and disseminated through relational assets. As a result, communication processes become an essential aspect. The development of "the needs of the present without compromising the ability of future generations to meet their own needs" can be accomplished through communication also [1]. Instead, it calls for social and organizational intelligence and adoption of a strategy that considers new models placing an emphasis on collaboration and interaction between individuals and groups. The decision about communication methods is influenced by cognitive variations [2]. Information technologies actually alter people’s mental attitudes from a very young age, liberating from "proxemic" elements; typically, "face to face" contact. If technology can influence potential channels through which there is social connectivity, it would be fascinating to investigate how social media can change the intentions of people. One of the requirements for changing one’s attitude and behavior towards the environment for mitigation of climatic changes and global warming is consciousness about environmental sustainability.

Regarding the promotion of environmental sustainability, there are two viewpoints regarding behavioral change. First view posits that behavioral changes occur when the public’s knowledge and attitude towards an issue are raised through awareness campaigns. The second viewpoint suggests that individuals can make decisions based on their economic self-interest after carefully examining their options, without necessarily having prior knowledge or awareness of the issue. Although it is recognized that the social marketing is extremely influential at promoting consistent behavior [3]. The earlier literature confirms that interventions to increase awareness can lead to change the behavior. The trans theoretical model explains that environmental sustainability awareness is a source of behavioral change [4–7], and empirical findings also support the trans theoretical model [8,9].

Social media’s influence has grown over the time where we now use it to spread news, promote elections, and even carry out corporate operations [10]. Traditional media has been replaced by social media as most popular form of communications because of how quickly and easily it can be used [11]. Additionally, compared to conventional communication platforms, social media is a trustworthy source of knowledge [12,13]. It is used to spread information about environmental preservation. When determining how sustainable a company or product is, consumers frequently turn to social media [14]. Social media, on the other hand, frequently serves as an excellent platform for businesses to inform customers about their environmental performance [15]. Schroeder et al. [16] and Redecker [17] are of view that the popularity and utility of social media is important for awareness regarding environment. Social media has become popular recently to foster interpersonal communications and team work [18,19]. Social media is an effective tool for quick communication and a medium to disseminate the information [20–22]. As a result, potential of social media platforms could be further investigated for preservation of the environment. Social media is therefore crucial for affecting the environmental consciousness of China’s Z generation.

Generation born between middle of the 1990s and middle of the 2000s are referred as members of the Z generation, or Gen Z. This generation in China is recognized to be more environmentally sensitive than previous generations since they have grown up with access to social media platforms [23]. In China’s Z generation, social media and environmental sustainability are related in the following ways: People can communicate knowledge about environmental problems and sustainable practices using social media platforms like WeChat, Weibo, and Douyin [24]. People in China’s Z generation utilize social media to learn about environmental issues and to keep up with news about sustainability-related activities. Second, the Chinese Z generation is renowned for being open to participating in online activism to promote environmental sustainability [25]. They use social media platforms to join petitions, share articles, and take part in online campaigns that promote sustainable practices and raise awareness of environmental issues. Third, brands that place a high priority on sustainability and environmental responsibility are more likely to get the support of China’s Z generation. Social media gives both businesses and customers a platform to exchange information about their sustainability activities and environmentally friendly goods and services. Fourthly, the Chinese Z generation uses social media to encourage sustainable habits such lowering meat consumption, utilizing public transit, and minimizing plastic waste [23]. They urge others to adopt similar behaviors by using social media to offer sustainable living advice, resources, and success stories. Fifthly, members of the Z generation are more likely to choose products that support the environment. Consumers can explore and compare environmentally friendly items on social media, as well as exchange feedback and suggestions. In general, social media has been quite effective in encouraging China’s Z generation to practice environmental sustainability. Social media increasing public awareness about environmental issues and promoting environmentally friendly attitudes and practices through information sharing, online activism, brand awareness, lifestyle promotion, and green consumerism [21].

With a focus on China’s Z generation, this article aims to determine how social media might be used to facilitate environmental preservation. Social media is opening new dimensions in study of human interaction with natural environment as more than half population of world is attached with social media [15]. Earlier literature has the absence of a comprehensive behavior change model that explains the mechanism through which social media influences sustainable behaviors among the Z Generation in China. A well-developed behavior change model would provide a clear framework for understanding the causal relationships and factors that drive individuals to adopt sustainable practices based on their social media usage. This study will address that how does social media exposure lead to increased awareness of environmental issues among the Z Generation? How do attitudes toward sustainability evolve through social media interaction? Does social media exposure lead to positive shifts in attitudes, and if so, how are these attitudes translated into actions? How do social media influence perceptions of social norms relate to sustainable behaviors? Are there trends in adopting certain behaviors due to perceived societal expectations? Several scholars have conducted extensive research on impact of social media on consumer behavior and purchasing intention, especially in food industry. The current study, however, focuses on how social media influences consumer perceptions and factors including green consumption habits, eco-branding, eco-labeling, green purchase intention among China’s Z generation. By evaluating the influence of social media on consumers’ behavior, intentions and subjective norms towards green consumption, the current research study will close a research gap. The research methodology of this study is established on the Theory of Planned Behavior regarding behavior of green consumption. The novelty of the study is examination of the ways in which social media has a directing and influencing role in purchase intention, eco-branding, eco-labeling, and consumption behavior.

## 2. Conceptual model and hypothesis

Green consumption, sometimes referred to as sustainable consumption, is the process of consciously and purposefully choosing to buy products and services that have a lower environmental impact [13]. This entails taking into account a product’s life cycle, from creation to dispose of, and choosing goods that are produced with a low carbon footprint, from renewable resources, and that are recyclable or biodegradable. As more individuals become conscious of the effects, their purchase decisions have on the environment, green consumption is growing in popularity. Nowadays, buyers are looking for items that are both environmentally and socially conscious. Companies are responding to this trend by launching sustainable products, including eco-friendly procedures into their manufacturing processes, and utilizing eco-labels to promote environmental responsibility [21]. Benefits of eating green are numerous. It encourages the growth of a sustainable economy, conserves natural resources, and aids in lowering the carbon footprint of people and businesses. Customers may push businesses to adopt more sustainable practices and lessen their influence on the environment by supporting green products. Long-term cost benefits can come from green consumption as many sustainable items are made to be long-lasting and energy-efficient [25], which can lead to cheaper maintenance and energy expenditures. Green consumption can be extremely important in lowering carbon emissions, one of the main causes of climate change. Transportation, industrial processes, and the use of fossil fuels as an energy source are only a few of the human activities that cause carbon emissions [18]. By encouraging renewable energy source, lowering energy consumption, and supporting sustainable practices, green consumption can aid in the reduction of carbon emissions. Promoting the renewable energy like hydro power, wind, and solar is one way that green consumption can lower carbon emissions [25]. By choosing to purchase goods and services from companies that use renewable energy, consumers support clean energy technologies [23]. People can further lower their carbon footprint by deciding to install solar panels or other renewable energy sources in their homes. By using less energy, green consumption can also cut carbon emissions [26]. Finally, green consumption can promote sustainable practices such as recycling and composting, which reduces the quantity waste.

According to Zafar et al. [26], "green purchase intentions" refers to consumers’ propensity or willingness to purchase goods or services that are ecologically friendly. Consumers that have green buying intents are driven by a desire to limit their influence on the environment, support sustainable practices, and promote social responsibility [27]. Consumers are more conscious about environmental effect of their shopping decisions and there is tendency to increase such consciousness. Green consumption is influenced by a number of things. The awareness of consumer and their knowledge about environmental degradation is one of the most crucial factors [28]. Consumers are more inclined to seek out goods and services that have a smaller environmental impact as they grow more knowledgeable about environmental issues like pollution and climate change [29].

**H1:** Green purchase intentions are significantly influenced by social media.

Companies that are open and honest about their environmental policies and the sustainability of their products can help to raise customer awareness and affect intentions of consumers for green consumption. The accessibility and affordability of green products is another aspect that affects green purchase intentions of consumers [30]. Even while consumers might be eager to buy ecologically friendly products, they might decide not to if they are hard to find or much more expensive than non-green alternatives. Green purchase intentions are influenced by social and cultural factors also [28]. Socially and ecologically concerned consumers may be impacted by the beliefs and actions of their peers as well as by the cultural values and conventions. Social and cultural influencers can encourage green purchase intentions among their followers by encouraging sustainable practices and increasing knowledge of environmental challenges [28].

**H2:** There is a significant impact of green purchase intentions on green consumption behavior.

Subjective norms are ideas and opinions about what close friends or family members believe a person should do in a specific circumstance. These significant individuals could be a person’s relatives, friends, coworkers, or other important persons in their life [28–30]. Subjective norms have significant impact to affect human behavior and choices, especially those pertaining to environmentally friendly consumption [31]. According to Tan et al. [27], subjective norms are divided into injunctive norms and descriptive norms. While descriptive norm refers to beliefs about what significant others actually do in a given scenario, injunctive norms refer to perceptions about what significant others think to be socially acceptable or desirable behavior. Subjective norms can have a variety of effects on consumer behavior when it comes to environmentally friendly purchase. For instance, a person may be more inclined to engage in green consuming behaviors if they believe that their family and friends respect ecologically friendly goods and methods. On the other hand, someone may be less likely to practice green consumption habits if they believe that their social circle does not place a high priority on ecology. Additionally, societal norms and cultural values may have an impact on subjective norms. For instance, strong social norms regarding environmentalism and sustainability may exist in some cultures, which can affect people’s green consumption patterns [32].

**H3:** There is a significant impact of subjective norms on green consumption behavior.

The moderating role of eco-labeling between green purchase intentions and social media refers to how the influence of social media on consumers’ intentions to make environmentally friendly (green) purchases is contingent upon the presence and effectiveness of eco-labels on products or services [11]. In other words, eco-labeling can either enhance or weaken the relationship between social media exposure and consumers’ intentions to buy environmentally sustainable products. Consumers who are environmentally conscious might be motivated to support eco-friendly products to contribute to environmental protection [21]. If eco-labeling effectively communicates a product’s sustainability features, it can strengthen the positive impact of social media exposure on consumers’ green purchase intentions [28]. In this case, social media can raise awareness, and eco-labels provide tangible evidence that aligns with the messages consumers encounter on social media [23]. Companies can advertise their ecologically friendly goods and procedures via eco branding and eco labelling [27]. Eco labelling entails the use of labels or certifications to show that a product has complied with specific environmental criteria. The moderating role of eco-labeling in the relationship between social media and green purchase intentions highlights the importance of clear, credible, and informative eco-labels [24]. Effective eco-labeling can reinforce the messages consumers receive through social media and enhance their intentions to make environmentally sustainable purchases, while inadequate eco-labeling can lead to skepticism and weaken the positive impact of social media exposure [28].

**H4:** There is moderating role of eco-labeling between green purchase intentions and social media.

The moderating role of eco-labeling between social norms and social media refers to how the presence and effectiveness of eco-labels on products or services can influence the relationship between social norms and individuals’ behavior or attitudes as shaped by their exposure to social media content [12]. Basically, social norms are unwritten rules or expectations that guide individuals’ behavior and attitudes based on the perceived beliefs and actions of others in a social group [15]. In the context of environmental sustainability, social norms might refer to the collective understanding that eco-friendly behaviors are desirable and expected. Effective eco-labeling can enhance the influence of positive social norms conveyed through social media [28]. When individuals encounter consistent messages about the desirability of eco-friendly behaviors on social media and also see clear and credible eco-labels on products, their inclination to follow those norms might increase. In this case, eco-labels serve as tangible evidence that reinforces the perceived social norms. If eco-labeling is inconsistent, confusing, or lacks credibility, it could weaken the influence of social norms promoted through social media [31]. Individuals might become skeptical about the alignment between the social norms they encounter online and the actual environmental attributes of products. Unclear or misleading eco-labels can cast doubt on the authenticity of the promoted social norms.

**H5:** There is moderating role of eco-labeling between social norms and social media.

Eco branding is the use of branding and marketing techniques to emphasize a firm’s devotion for environmental sustainability. Eco branding is a powerful strategy that businesses may use to stand out from rivals and attract customers that care about the environment [33]. Employing eco branding allows businesses to promote their use of sustainable products, carbon emission reduction efforts, and renewable energy sources. Companies can draw customers that value sustainability and could be willing to pay more for eco-friendly items by publicizing their environmentally friendly practices [34]. Another strategy firms use to market their ecologically friendly goods and procedures is eco labelling. Eco labels and certifications show that a product has complied with environmental requirements, such as using sustainable materials, avoiding toxic chemicals, or having a smaller negative effect on environment [35]. These labels can encourage consumers to trust in a firm’s environmental promises and assist consumers in making knowledgeable purchasing decisions. But it’s crucial to remember that not all eco labels are the same. While some labels are self-certified by the company, others may be supported by third-party certifications. Some labels are more stringent than others. To make wise purchasing decisions, consumers should be aware of the various eco label kinds and the principles they stand for [36].

**H6:** There is moderating role of eco-branding moderates between green purchase intentions and social media.

Social media is now a potent instrument for encouraging sustainable behaviors and increasing environmental awareness. Social media platforms, which have billions of users worldwide, offer a mechanism for people to interact, share information, and mobilize action on environmental issues [35,36]. Environmental issues like climate change, pollution, and habitat degradation can be brought to public attention using social media [27]. Individuals and organizations can contribute to public education and foster knowledge of these complicated issues by sharing news items, images, and videos pertaining to environmental challenges. Additionally, social media can be utilized to encourage environmentally beneficial practices including recycling, conserving energy, and using eco-friendly items [37]. Social media users can inspire others to embrace sustainable lifestyles and have a good impact on the environment by sharing sustainable living advice, resources, and success stories. Social media can be employed to encourage people to take action on environmental issues.

**H7:** Social norms are influenced by social media in a significant way.

Online petitions and activism can compel governments and businesses to take action on environmental issues, while social media campaigns and hashtags can increase awareness and support for environment [38]. It’s crucial to keep in mind, too, that disinformation and greenwashing can also be spread through social media. Social media can be used by certain people and organizations to spread incorrect or misleading information about environmental challenges or to exaggerate the benefits of their own sustainability efforts. To confirm the veracity of the content they encounter on social media, consumers should exercise caution and conduct their own research [39]. In conclusion, social media has developed into a potent instrument for encouraging sustainable behaviors and increasing environmental awareness. Social media users can help to create a more sustainable future by sharing knowledge, encouraging sustainable behaviors, and mobilizing action on environmental issues [40].

“An explanation of how people’s attitudes, subjective norms, and perceived behavioral control impact their intentions and behaviors is provided by the Theory of Planned Behavior (TPB), a social psychology theory” [40]. TPB highlights that intentions of individuals affecting human behavior are effected by subjective norms, perceived behavioral control, and attitudes. An individual’s assessment of the relevant behavior, either favorably or unfavorably. Beliefs about how a behavior will turn out, including expected rewards and costs, have an impact on attitudes [41]. Subjective norms are influenced by an individual’s motivation to conform to these ideas as well as beliefs about what important others think of the behavior. Beliefs about existence of facilitating or impeding elements, such as resources, skills, and opportunities, have an impact on perceived behavioral control. According to TPB, a person is more likely to carry out a behavior if their intentions to do so are stronger [42]. The theory does admit, however, that circumstances beyond a person’s control, such environmental restrictions, may influence their capacity to change the behavior [43]. A wide range of behaviors, including consumer, environmental, and health-related behaviors, have been explained using TPB [31]. TPB can help informing the design of interventions and campaigns targeted at encouraging desired behaviors and attitudes by understanding the factors that shape intentions and behaviors [43]. Green production, green consumption, and environmental sustainability are serious concerns and popular among consumers [44,45]. Attitudes of consumers and their abilities have evolved over the time and they now believe that green consumption is the primary driver of environmental preservation [29]. There is a significant change in consumption behaviors and patterns of modern consumers [38]. It is needed to explore the determinants influencing the behaviors of modern consumers regarding green consumption.

**H8:** Social media plays a positive role on green consumption behaviors.

The conceptual framework of the study is given in Fig 1.

**Fig 1:** Conceptual framework.

The practical implications underscore the role of social media in influencing consumer choices and shaping brand-consumer interactions. On the other hand, theoretical implications provide a framework for understanding the psychological mechanisms through which social media impacts green purchase behavior. Both aspects highlight the transformative potential of social media in driving more sustainable consumption patterns [31]. Social media provides a rapid and wide-reaching platform for sharing information about environmentally-friendly products, practices, and companies. This makes it easier for consumers to access information about green products and make informed purchasing decisions [34]. Moreover, social media empowers consumers by allowing them to share their experiences, reviews, and recommendations related to green products [28]. This peer-to-peer communication builds trust and credibility around sustainable purchases. In addition, brands are now more accountable due to the transparency demanded by social media. Consumers can use these platforms to scrutinize and hold companies accountable for their environmental claims and actions, influencing their purchasing decisions [35].

Theoretical implications of the study reveal that consumers often use social media to signal their identity and values [6]. The adoption of green products can become a way for individuals to express their commitment to environmental causes, aligning with their self-concept and social identity [15]. As per theory of planned behavior that social media exposure can influence consumers’ attitudes, subjective norms, and perceived behavioral control regarding green purchases. The continuous exposure to green content can shape their intention to buy eco-friendly products. The social learning theory also highlights that social media provides a platform for consumers to observe and learn from others’ behaviors [37]. Seeing peers make green choices and discussing the benefits can motivate individuals to adopt similar behaviors.

## 3. Materials and methods

The respondents were given a questionnaire that had been adopted in previous studies to accomplish the goals of the study. The written ethical consent was received from the respondents in the beginning then questionnaire was sent to those participants who were willing to participate in the study. Moreover, questionnaire was equipped with objectives and information of the study. China’s Z generation was the target population and convenience sampling method is adopted. This approach could be used for initial exploratory research or when convenience is a primary concern. The respondent is surveyed for cross-sectional data. The widely used scales in earlier literature are considered [46,47], and two experts in the field are consulted to omit any ambiguous entries to assure reliability and questionnaire validity. In addition, a pre survey of 50 samples is conducted to avoid any translation errors. After ensuring the error-free translation of the questionnaire, a complete sample is collected. The online resources like social media platforms are used to collect the data by using formal questionnaires. The random sampling procedure is adopted for collection of data. Those questionnaires were not considered in which participants did not match the requirements of the study. Those questionnaires were also excluded from the analysis, which found some ambiguities. Questionnaire was sent via social media to 650 individuals but 563 responses were selected for empirical analysis as remaining responses were not suitable for analysis. The questionnaires with missing values were eliminated throughout the screening process since, according to research, those with more than 10% of the values missing should not be taken into account. Similar to the above, 22 surveys were eliminated because of abnormalities, duplications, and outliers. The scales and sub constructs are shown in the Table 1.

**Table 1:** Scales and constructs.

**Social Media**
I use social media to interact with others regarding green products.
The information shared on social media influences the purchase of the green product.
I gain feedback on green products through environmental information on social media.
I trust information shared on social media regarding green products.
**Green Consumption Behavior**
I used to learn about green products.
I recommend green products to other people.
I prefer to purchase the green product.
The information shared on social media encourages me for purchasing of green products.
**Green Purchase Intentions**
Green products are better for the environment as compared with general products.
Green products have value against paid money.
I expect that green products increase environmental performance.
**Eco-Labeling**
I plan to purchase eco-labeled products in the future.
I am willing to purchase more eco-labeled products while shopping.
From now on, I plan to purchase eco-labeled products.
I intend to pay more for eco-labeled products.
**Eco-Branding**
For those brands that use green messages in their advertisements, I think they are good.
I take attention to eco-labeled products through green advertising.
Green advertising is valuable in my opinion.
**Subjective Norms**
I perceive that social development is associated with green products.
I perceive that family wishes are associated with green products.
I perceive that national policy is associated with green products.

### 3.1. Data analysis and findings

The demographic information and descriptive analysis are evaluated and analyzed in accordance with the research guideline. In Table 2, demographics are provided. The findings show that 563 people took part in the survey. The majority of respondents—68.38%—have bachelor’s degrees, followed by master’s degrees (26.70%), and PhDs (3.90%). Additionally, Table 2 includes general information about respondents.

**Table 2:** Demographic analysis (N = 563).

Item	Sub-Item	Frequency	Percentage
Education	Bachelor Level	385	68.38
	Master Level	156	27.70
	PhD Level	22	3.90
Gender	Male	308	54.71
	Female	255	45.29
Age	20–24 years	189	33.57
	25–29	296	52.56
	30–34	78	13.85
Usage experience of social media	1–4 years	204	36.23
	5–8	199	35.35
	9–12	160	28.42
Daily usage of social media	1–3 hours	178	31.62
	4–6	295	52.40
	7–9	90	15.98

After descriptive analysis, the internal consistency, convergent validity and reliability of the model is examined. In the initial steps, the composite reliability (CR) and Cronbach’s α (CA) are determined to find the internal consistency of the model and findings are shown in Table 3.

**Table 3:** Factor loadings.

Constructs	Factor loading	Cronbach’s α	Composite reliability	Average variance extracted
Social Media (SOM)		0.75	0.86	0.61
1	0.69			
2	0.72			
3	0.81			
4	0.88			
Green consumption behavior (GRB)		0.73	0.84	0.63
5	0.83			
6	0.75			
7	0.89			
8	0.90			
Green consumption intention (GRI)		0.75	0.83	0.66
9	0.79			
10	0.86			
11	0.64			
12	0.59			
Eco-labeling (ECL)		0.71	0.80	0.59
13	0.64			
14	0.69			
15	0.66			
16	0.65			
Eco-branding (ECB)		0.73	0.86	0.70
17	0.72			
18	0.69			
19	0.73			
Subjective norms (SBN)		0.86	0.83	0.67
20	0.89			
21	0.81			
22	0.77			
23	0.58			

The values of CR and CA are in range of accepted values as highlighted by Dhir et al. [29]. The value of CA lies between 0.71–0.86 indicating the good internal consistency of all items of the constructs. While the values of CR fall in range of 0.80–0.86 supporting the values of CA. In addition, factor loading is computed to determine convergent validity through “average variance extracted” (AVE). Each value of AVE is ˃ 0.5 showing the reliability of the model.

The discriminant validity is computed through many approaches but research studies prefer to apply Heterotrait Monotrait ratio of correlations (HTMT) and Fornell Lacker approaches to determine discriminant validity. Discriminant validity refers to the extent to which two different constructs or variables, which are theoretically distinct, are actually distinguishable from each other in a measurement or assessment context. In other words, discriminant validity assesses whether a measurement instrument can accurately differentiate between two or more concepts that should not be too highly correlated with each other. If the items that are supposed to measure different constructs load more heavily on their respective factors and less on other factors, this suggests good discriminant validity. The rule highlights that values of inter correlation among constructs should be less than the square root of AVE. The estimated values of discriminant validity are shown in Table 4 which conveys that model may be used for further analysis.

**Table 4:** Fornell larcker approach.

Construct	ECL	GRI	ECB	GRB	SOM	SBN
ECL	0.82					
GRI	0.56	0.77				
ECB	0.58	0.63	0.79			
GRB	0.51	0.57	0.59	0.87		
SOM	0.24	0.58	0.39	0.27	0.73	
SBN	0.23	0.44	0.49	0.55	0.38	0.85

ECL = Eco-labeling; GRI = Green consumption intention; ECB = Eco-branding; GRB = Green consumption behavior; SOM = Social media; SBN = Subjective norms.

Fornell Larcker approach is used to determine whether the latent variables or constructs in a research model are distinct from each other and can be reliably differentiated. The Fornell-Larcker approach involves conducting a CFA and analyzing the squared correlations (variances) between latent variables and their associated measurement indicators. In other words, if the squared correlation (shared variance) between two latent variables is smaller than both the variance extracted for each of those variables, then discriminant validity is supported. If this condition is not met, it might indicate potential issues with the distinctiveness of the latent variables, suggesting that further refinement of the measurement model may be needed.

Henseler et al. [48] devised the HTMT technique highlighting the discriminant validity. The (HTMT) ratio of correlations is also a statistical technique used to assess discriminant validity. It was proposed as an alternative method to evaluate discriminant validity compared to other methods. The HTMT ratio of correlations focuses on the idea that when assessing discriminant validity, the correlations between items measuring different traits (heterotrait correlations) should be smaller than the correlations between items measuring the same trait (monotrait correlations). In other words, if items that belong to the same construct (monotrait) have higher correlations with each other than items from different constructs (heterotrait), it suggests that the measurement instrument effectively differentiates between distinct constructs. The HTMT ratio can range from 0 to 1. A value of 0 indicates perfect discriminant validity (no overlap between constructs), while a value of 1 suggests that there is no discriminant validity (constructs are indistinguishable). In general, lower values of the HTMT ratio (closer to 0) are indicative of better discriminant validity. The values of HTMT are less than standard value of 0.90, as reported in Table 5.

**Table 5:** HTMT approach.

Construct	ECL	GRI	ECB	GRB	SOM	SBN
ECL						
GRI	0.47					
ECB	0.64	0.77				
GRB	0.63	0.71	0.73			
SOM	0.41	0.58	0.72	0.37		
SBN	0.30	0.59	0.46	0.58	0.34	

After finding the discriminant validity, researchers evaluate the structural model using PLS-SEM through six criteria [29]. The PLS-SEM model involves understanding the relationships between latent variables, their indicators, and the path coefficients representing these relationships. In the beginning, fitness of the model is assessed. Then path coefficients between latent variables are examined. These coefficients represent the strength and direction of the relationships between constructs. Positive coefficients indicate a positive relationship, while negative coefficients indicate a negative relationship. The magnitude of the coefficients indicates the relative strength of the relationships. If the t-value is above a certain threshold (often 1.96 for a 95% confidence level), the relationship is considered statistically significant. Higher R^2^ values suggest that the model is better at explaining the variance in the construct. The factor loadings indicate how well the indicators represent the latent variables. Larger loadings indicate stronger relationships between indicators and latent variables. The issue if multicollinearity is addressed in the first stage. Similarly, “assessing the amount of impact size (f2), the level of effect size (R2), and the predictive significance of the structural model relationship is important for determining the relationship’s importance (Q2). Furthermore, using bootstrapping with 5000 resamples, it is crucial to evaluate the corresponding *t*-values of the path coefficients. The evaluation of the relationship’s impact sizes is crucial because the *p*-values only informs us of the existence of an effect but not its magnitude” [47]. Table 6 contains the results of R^2^, F^2^, VIF, and Q^2^.

**Table 6:** Structural model.

R^2^	Dependent variable GRB	R^2^ 0.35	R^2^ adjusted 0.34	Gong et al. [37] 0.02 = weak 0.13 = moderate 0.26 = substantial
F^2^	Independent variables		Green consumption	
	ECL			
	GRI		0.101	
	ECB			
	GRB	0.036	0.110	
	SOM	0.050	0.040	
	SBN	0.001	0.006	
Inner VIF	Independent variable		GRB	VIF ≤ 5.0
	ECL	1.43	2.10	
	GRB	1.38		
	GRI	2.54	2.71	
	ECB	2.79	2.36	
	SOM	2.96	2.83	
	SBN	2.91	1.69	
Q^2^ = 1-SSE/SSO	Dependent variable	CCR	CCC	
	GRI	0.19	0.53	
	GRB	0.23	0.56	
	SBN	0.21	0.54	

CCR = “constructs cross-validated redundancy”; CCC = “constructs cross-validated communalities”.

All values are in acceptable range so all hypotheses may be accepted. The values of LCL and UCL are positive while T and P values are significant as shown in Table 7.

**Table 7:** Path coefficients.

Hypotheses	β/OS	LL	UL	T	P
ECL ➝ GRI	0.14	0.13	0.31	0.95	0.02
GRI ➝ GRB	0.41	0.15	0.59	2.98	0.01
ECB ➝ GRI	0.39	0.17	0.63	2.51	0.01
SOM ➝ ECL	0.28	0.04	0.51	2.39	0.00
SOM➝ GRI	0.33	0.11	0.58	3.11	0.00
SOM ➝ ECB	0.39	0.07	0.44	2.95	0.00
SOM ➝ GRB	0.21	0.38	0.26	1.93	0.01
SOM ➝ SBN	0.26	0.05	0.41	2.01	0.03
SBN ➝ GRB	0.39	0.16	0.59	2.99	0.01

The constructs in Table 7 demonstrate how social media has an impact on intentions of consumers regarding green consumption. The general public is returning to green consumption, as indicated in earlier literature; this is also confirmed by findings of this study. The values of the mediating effect confirm the results of the direct hypotheses. It shows that social media is effectively controlling and influencing the intentions and behaviors of consumers regarding green consumption. The analysis of the study has confirmed that social media is actively involved in altering and influencing consumer behaviors towards a preference for environmentally friendly consumption. The hypothesis of mediation is also supported, as the values fall within the accepting range, with no negative values observed for any construct for the lower or upper limit. The results of the mediation analysis are shown in Table 8.

**Table 8:** Mediation analysis.

Hypothesis	β/OS	LL	UL	T	P
SOM ➝ ECL ➝ GRI	0.02	0.03	0.14	0.91	0.29
SOM ➝ ECB ➝ GRI	0.13	0.01	0.29	1.39	0.11
ECL ➝ GRI ➝ GRB	0.04	0.07	0.17	0.77	0.32
SOM ➝ ECL ➝ GRI ➝ GRB	0.22	0.07	0.04	0.63	0.38
ECB ➝ GRI ➝ GRB	0.15	0.05	0.46	1.93	0.04
SOM ➝ ECB ➝ GRI ➝ GRB	0.06	0.10	0.16	1.71	0.21
SOM ➝ GRI ➝ GRB	0.15	0.04	0.33	1.98	0.04
SOM ➝ SBN ➝ GRB	0.12	0.19	0.13	1.81	0.05

### 3.2. Path coefficient (indirect effect) result

The sign of the path coefficient indicates the direction of the relationship between the variables. A positive coefficient implies a positive association, while a negative coefficient suggests a negative association. The magnitude (absolute value) of the path coefficient indicates the strength of the relationship. Larger coefficients indicate stronger relationships, while smaller coefficients indicate weaker relationships. Path coefficients are often accompanied by t-values or bootstrap confidence intervals. A coefficient is considered statistically significant if its t-value is larger than a critical threshold (e.g., 1.96 for a 95% confidence level). Non-significant coefficients may indicate that the relationship between the variables is not robust. Additionally, the “factor loading” and “convergent validity” using AVE supported the findings of the study. The values of constructs are compared to their comparable inter-correlation values, and the measurement model is in a position to move forward with the subsequent processes stated in Table 9.

**Table 9:** Path coefficients (indirect effect).

Hypotheses	β/OS	LL	UL	T	P
ECL ➝ GRI	0.11	0.13	0.32	0.54	0.02
GRI ➝ GRB	0.42	0.12	0.69	2.75	0.03
ECB ➝ GRI	0.35	0.07	0.61	2.63	0.01
SOM ➝ ECL	0.27	0.03	0.42	2.56	0.01
SOM ➝ GRI	0.35	0.16	0.55	2.88	0.01
SOM ➝ ECB	0.31	0.09	0.49	2.29	0.03
SOM ➝ GRB	0.19	0.35	0.16	1.69	0.01
SOM ➝ SBN	0.21	0.04	0.35	1.91	0.02
SBN ➝ GRB	0.37	0.14	0.47	2.62	0.00

Along with direct hypothesis that social media is positively influencing consumer intention and green consumption behavior, the mediating impact is also examined. As values are in acceptable range, the mediation hypothesis is accepted; as a result, social media is persistent in the study analysis. The study’s key findings imply that the entire working and learning process, as well as the social media and digital transformation era, have changed.

## 4. Discussion

The objectives of this study are to determine the influencing mechanism of social media on green consumption of Z generation of China. The findings demonstrate that social media significantly affects patterns of consumption. It is not unexpected that the entire working and learning mechanism has altered in the age of digital transformation, and social media has been rated as one of the best companions for young people [18]. The majority of nations make use of social media platforms to persuade and influence the general population, particularly young people, to adopt positive behaviors [23]. The findings of the study reveal that social media has a statistical positive significant relationship with green purchase intentions. Social media platforms provide a space for sharing information about eco-friendly products, sustainable practices, and their benefits [37]. Consumers can learn about the environmental impact of different products and make more informed decisions based on the information they gather. Moreover, social media allows users to observe and interact with peers, influencers, and brands that promote sustainable lifestyles [41]. As sustainable behavior becomes more normalized in these online communities, individuals may be motivated to align their own behaviors with those of the people they follow. Personal recommendations and testimonials from friends, family, and online influencers can carry significant weight [22]. Positive reviews and experiences shared on social media can positively impact consumers’ perceptions of green products and encourage them to consider making similar choices. It is also found that young generation is more careful about environmental sustainability. According to a survey by Nielsen, 68% of Chinese consumers in their 20s and 30s are willing to pay more for environmentally-friendly products, and 46% of them are actively seeking out eco-friendly products [29]. Social media is playing a crucial role in this shift towards green consumption. In addition, social media has also made it easier for consumers to access information about eco-friendly products and compare prices and features. E-commerce platforms like Tmall and JD.com have also introduced eco-friendly product categories, making it easier for consumers to find and purchase green products [48]. The widespread focus on environmental issues has boosted organizations’ adoption of green business practices. It’s crucial for producers to comprehend the elements influencing the adoption of green consumption as well as the benefits of green production and consumption. This research is creating a sarcastic and emotive model of green consumption, which is an essential initial step for any upcoming profound comprehension [49].

The study depicts that subjective norms have a significant impact on green consumption behavior. In the context of green consumption, subjective norms relate to how much an individual feel that their friends, family, peers, or society expects them to engage in environmentally-friendly behaviors [39]. People tend to conform to the expectations and behaviors of their social groups. If an individual perceives that their peers or social network values and practices green consumption, they are more likely to adopt similar behaviors to fit in or gain approval [27]. Subjective norms are influenced by an individual’s beliefs about what others think they should do. If an individual believes that their friends and family value eco-friendly choices, they are more likely to internalize those beliefs and align their consumption behavior accordingly [36]. If an individual observes their peers making environmentally-conscious choices, they may feel motivated to do the same to maintain a positive self-image or to avoid standing out negatively [41].

The study found that eco-branding and eco-labelling act as moderating factors that influence the relationship between green purchase intentions and social media in the context of environmentally-friendly consumer behavior. When a brand emphasizes its commitment to sustainability, it can enhance consumers’ perceptions of the brand’s credibility and authenticity in promoting eco-friendly products [26]. This can moderate the relationship between green purchase intentions and social media in several ways. If a brand with strong eco branding promotes green products on social media, consumers are more likely to perceive the information as trustworthy and reliable [32]. This can lead to a stronger influence of social media content on consumers’ green purchase intentions [42].

Eco-labelling involves the use of labels or certifications to indicate a product’s environmental attributes and adherence to specific sustainability standards [26]. When consumers see such labels, they infer that the product meets certain ecological criteria [45]. Eco-labelling provides clear, standardized information about a product’s eco-friendliness. When this information aligns with messages on social media, it can reinforce the credibility and accuracy of the information, making consumers more confident in their intentions to purchase green products [19]. In concluding, both eco branding and eco labelling can enhance the influence of social media on green purchase intentions by providing credibility, trust, consistency, and assurance.

We contend that an organization’s level of environmental and socioeconomic assertiveness affects the amount to which environmental and socioeconomic management strategies are implemented. Due to this, a rising number of financial institutions now acknowledge that a company’s involvement in the environment is a part of its corporate social responsibility [50–52]. A third reason that motivates businesses to practice corporate social responsibility is the denial of climate change [28,49]. On the other hand, prior research has a strong focus on the commercial sector [37]. According to our knowledge, this study is the first to examine how socioeconomic and environmental management are integrated across the banking sector as a whole. There is additional study that examines other outcomes, including socioeconomic performance and the environment, which are interconnected. To gain a competitive edge, for instance, organizational components, proactive behavior, and environmental attitudes must all be interconnected [35,42,53].

## 5. Conclusions

This study for the Chinese Z generation looks at the rising tendency towards eco-friendly consumption and the function of social media. In order to better understand the intentions behind green purchases and the behaviors associated with them, constructs are incorporated in the study. To further evaluate the context of the green consumption intentions and behaviors, subjective norms, objective norms, and personal preferences and experiences might be incorporated. Although the study advised trying the model in other developing and developed countries’ organizational and governance environments, more research can be done based on the limitations highlighted in the earlier section. In a similar vein, green consumption habits are being supported by an emerging field called artificial intelligence. As a result, comparative research may be carried out between diverse nations and cultural contexts, giving a wider perspective and enhancing the notions of green consumerism. Finally, the proposed model can be expanded in future study to incorporate green CSR accountability, competitive advantage, sustainability, and performance. Major findings of the study reveal that social media and digital transformation influence the general population, promising to give new directions to the behaviors. Additionally, the mediating effect was also examined because their values fall within the acceptable range. It can be concluding that the social media is one of the most influential sources in influencing consumer behaviors toward green consumption whereas the values of the UCL and LCL are positive.

The end-users’ consumption patterns are significantly changed, chained, and influenced by social media. Due to pandemics, the public is aware of their health, and various economies use social media platforms to persuade and influence the public. The development of the model of green consumption, a necessary first step for any future thorough comprehension, is the outcome of significant focus being placed on the environmental challenges that increased enterprises’ adoption of green business. This resulted in the development of institutional tools for evaluating the application of environmental management systems.

Despite a number of limitations, the researchers may use the study’s conclusions as a road map for the field of green consumption. Using a conceptual framework, future research may examine how environmental management system affect the use of ecological performance metrics. When developing and implementing an approach, external contextual components are connected to internal components [31,53]. The effectiveness of environmental management system may be assessed using institutional measures.

## Supporting information

S1 Data (XLSX)
